# Long Noncoding RNA SAMMSON Promotes Melanoma Progression by Inhibiting FOXA2 Expression

**DOI:** 10.1155/2023/8934210

**Published:** 2023-02-07

**Authors:** Lijuan Yang, Meiling Zhou, Shulei Wang, Xiaojia Yi, Guohang Xiong, Jing Cheng, Buqing Sai, Qiao Zhang, Zhe Yang, Yingmin Kuang, Yuechun Zhu

**Affiliations:** ^1^Department of Biochemistry and Molecular Biology, School of Basic Medical Sciences, Kunming Medical University, Kunming, China; ^2^Department of Pathology, School of Basic Medical Sciences, Kunming Medical University, Kunming, China; ^3^Department of Student Affairs, Guilin University of Technology Nanning Branch, Nanning, China; ^4^Department of Pathology, The Second Affiliated Hospital of Kunming Medical University, Kunming, China; ^5^Department of Pathology, The First Affiliated Hospital of Kunming Medical University, Kunming, China; ^6^Department of Organ Transplantation, The First Affiliated Hospital of Kunming Medical University, Kunming, China

## Abstract

Long noncoding RNAs (lncRNAs) play crucial roles in melanoma initiation and development, serving as potential therapeutic targets and prognostic markers for melanoma. lncRNA survival-associated mitochondrial melanoma-specific oncogenic noncoding RNA (SAMMSON) is upregulated in many types of human cancers. However, the functions of SAMMSON in melanoma have not been fully elucidated. This study is aimed at investigating the expression and functions of SAMMSON in melanoma development. Bioinformatics analysis was performed to determine the expression of SAMMSON and its correlation with the 10-year overall survival (OS) in melanoma patients. Cell proliferation, migration, invasion, and tumorigenesis were detected by MTT, colony formation, Transwell assays, and mouse xenograft model. The expression of cell cycle-related factors, epithelial-to-mesenchymal transition (EMT) makers, and matrix metalloproteinases (MMPs) was assessed by RT-qPCR and western blotting analysis. The results demonstrated that SAMMSON expression was upregulated in melanoma tissues and cells, and lower SAMMSON expression was correlated with longer 10-year OS. SAMMSON knockdown decreased the proliferation, migration, and invasion of melanoma cells by regulating the expression of proliferation-related genes, EMT factors, and MMPs, respectively. Additionally, Forkhead box protein A2 (FOXA2) was confirmed to be a target of SAMMSON, and the biological effects induced by FOXA2 overexpression were similar to those induced by SAMMSON silencing in melanoma cells. Further studies showed that SAMMSON downregulated FOXA2 expression in melanoma cells by modulating the EZH2/H3K27me3 axis. Taken together, our data indicate that SAMMSON plays an important role in melanoma progression and can be a valuable biomarker and therapeutic target in melanoma.

## 1. Introduction

Malignant melanoma (MM) is the most aggressive form of skin cancer, and its incidence is increasing worldwide [1]. Treatments for MM have improved significantly over the years using targeted therapies and immune checkpoint inhibitors [2]. However, the benefits of these therapeutic modalities to patients with melanoma depend on the type and status of oncogene mutation. For instance, BRAF inhibitors mainly benefit patients with melanoma carrying *BRAF* mutations but not patients with other mutation types. In addition, the mutation status of the *BRAF* gene varies across populations [3], and *BRAF* mutational heterogeneity is common in melanomas [4]. These characteristics also explain differences in the clinical outcomes of melanoma treatment. Therefore, it is crucial to identify new and effective therapeutic targets and elucidate the mechanisms underlying melanoma progression.

lncRNAs are endogenous RNA molecules with more than 200 nucleotides and little or no coding potential [5]. Several lncRNAs associated with MM have been identified [6] and play an important role in melanoma growth and progression [7]. Moreover, the expression profile of lncRNAs is cell and tissue specific, making them attractive therapeutic targets and prognostic markers [8, 9].

Survival-associated mitochondrial melanoma-specific oncogenic noncoding RNA SAMMSON, located on chromosome 3p13-3p14, is ubiquitously expressed in human melanomas [10]. SAMMSON maintains melanoma cell survival by affecting mitochondrial function and translation processes by binding to different proteins, including P32, XRN2, and CARF [10, 11]. However, the role of SAMMSON in melanoma development is unclear.

FOXA2, a transcription factor (TF) of the FOXA family, is involved in tumor initiation and progression. For instance, in lung cancer, FOXA2 silencing induces tumor cell growth and survival by inhibiting apoptosis and promoting cell proliferation [12]; in turn, FOXA2 overexpression suppresses tumor cell migration, invasion, and EMT [13]. FOXA2 is downregulated in melanoma and suppressed melanoma cell proliferation and migration [14].

This study investigated the function of SAMMSON in melanoma progression and the underlying mechanisms. These findings provide insight into the regulation of melanoma proliferation, migration, and invasion.

## 2. Materials and Methods

### 2.1. Ethics Statement

The studies involving human participants were reviewed and approved by the Research Ethics Committee of Kunming Medical University (Grant No. KMMU2021MEC139). The use of the specimens was approved by the Institutional Review Board of the Third Affiliated Hospital of Kunming Medical University. All patients and their families gave written informed consent to use their tissue samples in accordance with the Declaration of Helsinki [15]. All animal experiments were approved by the Animal Care and Use Committee of Kunming Medical University.

### 2.2. Inclusion and Exclusion Criteria

The inclusion criteria were age > 18 years, patients with melanoma diagnosed histologically, patients with complete medical records, patients who volunteered and gave written informed consent, and patients with good compliance and long-term follow-up.

The exclusion criteria were patients with severe acute infections or autoimmune diseases, patients with a history of other malignancies, and patients who underwent chemoradiotherapy.

### 2.3. Melanoma Tissue Microarray

The tissue microarray MME1004i containing 67 human malignant melanoma tissues and 11 nevi tissues was purchased from Alenabio Biotech Co., Ltd (Xi'an, China). Patients were staged according to the American Joint Commission on Cancer (8th edition) classification criteria. The clinicopathological characteristics of our cohort are shown in Table 1.

### 2.4. Immunohistochemistry

Paraffin-embedded tissue sections were dewaxed in xylene and rehydrated in graded ethanol (2 × 10 min in absolute ethanol, 2 × 10 min in 95% ethanol, 1 × 10 min in 90% ethanol, 1 × 10 min in 85% ethanol, and 1 × 10 min in 70% ethanol) and ultrapure water. Heat-mediated antigen retrieval was performed using Tris-EDTA buffer pH 9.0 (Maxim, MVS-0099). Endogenous peroxidase activity was blocked with 3% hydrogen peroxidase in methyl alcohol for 10 min. Samples were incubated with primary monoclonal rabbit anti-FOXA2 antibody (1 : 100, ab108422, Abcam) overnight at 4°C and secondary goat anti-rabbit horseradish peroxidase-conjugated antibody (DAKO) for 1 h at room temperature. Tissue specimens were stained with diaminobenzidine and counterstained with hematoxylin.

The expression level of FOXA2 was independently and blindly evaluated by two pathologists based on the immunoreactive score (IRS) according to Remmele and Stegner [16]. Six fields of view near the tumor were randomly selected. The number of positive cells in each field was counted at 20x magnification, and the averages were calculated. Cells with a brownish-yellow color in the cytoplasm or nucleus were considered positively stained. Staining intensity was scored as 0 (negative), 1 (weak), 2 (moderate), and 3 (strong). The percentage of positive cells in each field of view was scored as 0 (0–5%), 1 (6–25%), 2 (26–50%), 3 (51–75%), and 4 (76–100%). The IRS (ranging from 0 to 12) was obtained by multiplying these two scores and was classified as negative (0 points), weak (1-4 points), moderate (5-8 points), and strong (9-12 points). For statistical analysis, scores of 0–4 and 5–12 were regarded as low and high expression, respectively.

### 2.5. Analysis of Human Cancer Databases

Melanoma datasets from the Gene Expression Profiling Interactive Analysis (GEPIA) (https://gepia.cancer-pku.cn), The Cancer Genome Atlas (TCGA) portal (http://tcga-data.nci.nih.gov), and the Gene Expression Omnibus (GEO) repository (https://www.ncbi.nlm.nih.gov/geo) were analyzed. The clinicopathologic parameters of patients from these GEO datasets are listed in Table 2.

### 2.6. Cell Lines and Cell Culturing

Human melanoma cell lines (SK-MEL-110, A375, A875, SK-MEL-28, and M21), human renal carcinoma cell lines (ACHN, CaKi-1, and 786-O), the immortalized human keratinocyte cell line HaCaT, and the proximal tubule epithelial cell line HK-2 were purchased from the Cell Bank of the Chinese Academy of Medical Science (Beijing, China) and cultured in Dulbecco's modified Eagle's medium (DMEM, Gibco, Thermo Fisher Scientific) supplemented with 10% fetal bovine serum (HyClone, Thermo Fisher Scientific) at 37°C in a humidified atmosphere of 5% CO_2_.

Cells were cultured in T-25 flasks until 85% confluence. Cells in the logarithmic growth phase were washed with phosphate-buffered saline (PBS) three times, detached by treatment with 0.05% trypsin, and washed with DMEM complete medium to inactivate trypsin. After that, the cells were harvested, pelleted by centrifugation, suspended in complete medium, stained with trypan blue (Sigma-Aldrich), and then counted using a TC20 automated cell counter (Thermo Fisher Scientific). Cells were plated on 6-well plates at a density of approximately 3.0 × 10^5^ per well for gene silencing studies, RNA isolation, protein extraction and flow cytometric assay and at 1.0 × 10^5^ per well for lentivirus infection assay. One day after plating, the cells were subjected to different treatments.

### 2.7. Gene Silencing and Establishment of Stable Cell Lines

Locked nucleic acid-modified antisense oligonucleotide (ASO), which trigger RNase H-mediated degradation of the target gene, were used to knock down lncRNA expression. Two SAMMSON-targeting ASOs (ASO 3 (GapmeR3), GTGTGAACTTGGCT and ASO 11 (GapmeR11), TTTGAGAGTTGGAGGA) previously validated by Leucci et al. [10] and a nontargeting ASO (TCATACTATATGACAG) were purchased from Exiqon. Transfection was performed using the Lipofectamine RNAiMAX transfection reagent (Cat. No. 13778075, Invitrogen; Carlsbad, CA, USA) according to the manufacturer's instructions. Briefly, early passage A375 and A875 cells were plated in 6-well plates at a density of approximately 2.0 × 10^5^ cells per well. In each well, 1 ml Opti-MEM medium (Cat. No. 11058021, Thermo Fisher Scientific) containing 2.5 *μ*l GapmeR (50 *μ*M) and 5 *μ*l Lipofectamine RNAiMAX transfection reagent were added to the cell culture. Cells were incubated with the transfection mixture for 16 h, and the medium was replaced with DMEM complete medium without antibiotics. Cells were harvested at 48 h for total RNA extraction and gene expression analysis and at 72 h for protein extraction.

To establish cell lines stably expressing FOXA2, 1.0 × 10^5^ A375 and A875 cells were plated into 6-well plates. On the next day, A375 and A875 cells were infected with FOXA2-overexpression (OE) lentivirus or a negative control (NC) overexpression lentivirus, respectively, in the presence of Hitrans G reagent (GeneChem). After 3 days, lentivirus-transduced cells were selected using 1.0 *μ*g/ml puromycin for approximately 21 days to generate stable FOXA2-OE melanoma cells and then continuously cultured with 0.5 *μ*g/ml puromycin. Stable cell lines were identified by RT-qPCR, and the expression levels of FOXA2 were quantified by western blotting.

### 2.8. Immunofluorescence Staining

Melanoma cells were grown on a Lab-Tek chambered cover glass (Thermo Fisher Scientific, Rochester, NY) at a density of 3.0 × 10^4^ cells per chamber. For immunofluorescence labeling, cells were fixed with 4% paraformaldehyde for 20 min at room temperature, permeabilized with 0.1% Triton X-100 in PBS on ice for 15 min, and blocked with 5% bovine serum albumin (BSA) at room temperature for 1 h. Cells were incubated with anti-mouse FOXA2 antibody (1 : 100, ab108422, Abcam) overnight at 4°C and with Cy3-conjugated sheep anti-mouse IgG antibody (1 : 100, Cat. No. C2181; Sigma-Aldrich) for 1 h at room temperature. After three washes with PBS, the cells were mounted with Fluoroshield with 4′,6-diamidino-2-phenylindole (Cat. No. F6057, Sigma-Aldrich) and imaged on an Olympus Fluoview laser scanning confocal microscope (Tokyo, Japan).

### 2.9. Cell Proliferation Assay

Melanoma cell proliferation was evaluated using the CellTiter 96 AQueous One Solution Cell Proliferation Assay (Cat. No. G3580; Promega, Fitchburg, WI, USA), according to the manufacturer's instructions. Cells were seeded into 96-well plates at 4.0 × 10^3^ cells per well with 200 *μ*l DMEM complete medium and cultured at 37°C in a humidified incubator with 5% CO_2_. Then, 20 *μ*l MTS reagent was added to each well at 0, 24, 48, 72, and 96 h after cell plating. The plates were incubated at 37°C for 4 h, and the absorbance was measured at 490 nm using an Infinite 200 PRO microplate reader (Tecan, Mannedorf, Switzerland).

### 2.10. Colony Formation Assay

Melanoma cells were subjected to different treatments and plated into 6-well plates at a density of 2.0 × 10^3^ cells per well. The culture medium was changed every 3 days. After 14 days, the cells were washed with PBS three times, fixed with 4% paraformaldehyde for 20 min at room temperature, stained with 0.5% crystal violet for 15 min at room temperature, and counted under a stereomicroscope.

### 2.11. Cell Cycle Analysis

Cell cycle analysis was performed by flow cytometry. Briefly, melanoma cells subjected to different treatments were trypsinized into single-cell suspensions, harvested, and pelleted by centrifugation. After washing with PBS three times, the cells were fixed with 70% cold ethanol overnight at 4°C. After two washes with PBS, fixed cells were suspended in PBS containing 1 mg/ml RNase (Sigma-Aldrich, St. Louis, MO, USA), incubated at 37°C for 1 h, and stained with 200 *μ*g/ml propidium iodide (Sigma-Aldrich) for 15 min at 4°C. DNA content was assessed by flow cytometry (FACSCelesta; BD Biosciences, USA) using ModiFit LT software version 3.2.

### 2.12. RT-qPCR

PCR was carried out using SYBR Green Master Mix (ROX) (#04913914001; Roche) following the manufacturer's instructions. The primer pairs were designed using Primer 3 software version 1.0 and are listed in Table 3.

Total RNA was extracted using TRIzol reagent (Cat. No. 9109; Takara) following the manufacturer's protocol. The RNA concentration was quantified using a Nanodrop spectrophotometer (ND1000; Thermo Fisher Scientific). RNA (2 *μ*g) was reverse transcribed to complementary DNA (cDNA) using the SuperScript III First-Strand Synthesis System (Cat. No 18080-051; Invitrogen) according to the manufacturer's instructions. Amplification was carried out in a 20 *μ*l reaction volume containing 10 *μ*l 2× SYBR Green Fast Master Mix (Invitrogen), 1 *μ*l of each primer (6 *μ*M), and 1 *μ*l of cDNA. PCR was performed using an ABI 7900HT Fast Real-Time PCR system (Applied Biosystems, USA). The amplification conditions consisted of an initial denaturation step at 95°C for 15 min, followed by 45 cycles at 94°C for 15 s, 60°C for 25 s, and 72°C for 20 s. The expression level of each target gene was normalized to the *β*-actin gene using the 2^–*ΔΔ*Ct^ method.

### 2.13. Western Blotting Analysis

Cells were washed twice with cold PBS and lysed with the M-PER Mammalian Protein Extraction Reagent (Cat. No. 78501; Thermo Fisher Scientific) and a protease inhibitor cocktail (Cat. No. 78410, Thermo Fisher Scientific). The lysate was collected by centrifugation at 12,000 rpm for 15 min at 4°C. Protein was quantified using a protein assay kit (Cat. No. 500-0002; Bio-Rad). Protein samples (80 *μ*g) were separated by sodium dodecyl sulfate-polyacrylamide gel electrophoresis and transferred to polyvinylidene difluoride membranes using a semidry electrophoretic transfer cell (Bio-Rad). The membranes were blocked with 5% nonfat milk or 5% BSA for 1 h at room temperature and incubated with anti-rabbit FOXA2 (1 : 1000; Cat. No. 8186; Cell Signaling Technology), anti-mouse MMP9 (1 : 1000; Cat. No. 13667; Cell Signaling Technology), anti-rabbit MMP2 (1 : 1000; Cat. No. 40994; Cell Signaling Technology), anti-rabbit GAPDH (1 : 5000; Cat. No.10494-1; Proteintech), and anti-mouse *β*-actin (1 : 10,000; Cat. No. A5441; Sigma-Aldrich) antibodies overnight at 4°C. The membranes were washed three times with 0.1% Tween in TBS and incubated with a horseradish peroxidase-conjugated secondary antibody for 1 h. Immunoreactive bands were visualized using the Super Signal West Pico chemiluminescent substrate detection system (Cat. No. 34077; Pierce Biotechnology). Fluorescence intensity was quantified using ImageJ software (National Institutes of Health). GAPDH and *β*-actin were used as loading controls.

### 2.14. Cell Migration and Invasion Assays

Cell migration and invasion were assayed with a Transwell system containing 8.0 *μ*m pores (Cat. No. 3428; Costar, Cambridge, MA, USA). Cells in the logarithmic growth phase were synchronized by serum starvation overnight. For cell invasion assays, transwell inserts were coated with 50 *μ*l of a mixture of serum-free DMEM and Matrigel (1 : 10, Cat No. 356234; BD Biosciences). After Matrigel solidification at 37°C for 4 h, synchronized cells (1 × 10^5^) in 200 *μ*l serum-free DMEM were seeded on the upper chamber and allowed to settle for 20 min, and 600 *μ*l of complete DMEM medium was added to the lower chamber. For the cell migration assay, synchronized cells (3.0 × 10^4^) were seeded on the upper chamber. Cells were incubated in a humidified incubator with 5% CO_2_ for 22 h (migration assay) or 36 h (invasion assay) at 37°C. After incubation, the medium in the Transwell chamber and outer wells was aspirated. The cells that migrated to the lower chamber were washed with PBS three times, fixed with 4% paraformaldehyde for 15 min, and stained with 0.1% crystal violet at room temperature for 30 min. The number of cells that migrated through the pores or invaded the Matrigel was counted. Cells in five representative fields were counted in each membrane.

### 2.15. Animal Experiments

All animal experiments were performed in accordance with the National Institutes of Health Guidelines for the Care and Use of Laboratory Animals [17]. Experimental procedures were approved by the Institutional Review Board of Kunming Medical University. Female BALB/C nude mice (4 to 6 weeks old) were obtained from the Animal Research Center of Kunming Medical University and maintained under specific pathogen-free conditions. For the *in vivo* proliferation assay, A375 NC-OE cells (transfected with a control vector) or A375 FOXA2-OE cells (5.0 × 10^6^ cells) were suspended in PBS and subcutaneously injected into the right flank of mice (five animals per group). Tumor volumes were monitored every 3 days. Tumor size was measured at different days postinjection using a Vernier caliper and expressed as volume (mm^3^) according to the formula: tumor volume = (length × width^2^)/2. Three weeks after injection, the animals were sacrificed by euthanasia, and tumors were excised and weighed.

### 2.16. Statistical Analyses

Statistical analysis was performed using SPSS version 20.0. The data are expressed as the mean ± standard deviation. The correlation between IRS and the clinicopathological features of each patient was analyzed using Fisher's exact test. Comparisons of two and more than two groups in *in vitro* experiments were performed using unpaired *t*-test and one-way analysis of variance, respectively. Differences were deemed significant when *p* < 0.05.

## 3. Results

### 3.1. SAMMSON Is Highly Expressed in Melanoma Tissues and Cells, and SAMMSON Upregulation Is Correlated with Shorter Survival

The expression of SAMMSON in melanoma and normal tissue was determined by analyzing the GEPIA database. SAMMSON expression was higher in melanoma tissues than in normal tissues (Figure 1(a)). The analysis of the GEO dataset revealed that SAMMSON expression was considerably greater in metastatic tissues than in normal skin and primary melanomas (Figure 1(b)). Furthermore, the analysis of the TCGA database showed that SAMMSON expression was higher in metastatic melanomas than in primary melanomas (Figure 1(c)).

SAMMSON expression was evaluated by RT-qPCR in melanoma tissues and cell lines. SAMMSON levels were significantly higher in melanoma tissues than in normal tissues in 80.0% (4/5) of cases (Figure 1(d)). In addition, relative SAMMSON expression increased in melanoma cell lines (A375, A875, SK-MEL-28, and M21) but not in renal carcinoma cell lines (ACHN, CaKi-1, and 786-O) or the non-tumorigenic cell lines HaCaT and HK-2 (Figure 1(e)). Log-rank analysis showed that 10-year OS was shorter in melanoma patients from the high SAMMSON expression group (Figure 1(f)). These data indicated that SAMMSON was highly expressed in melanoma tissues and cells, and that its upregulation could predict poor survival in patients with MM.

### 3.2. SAMMSON Knockdown Reduces Melanoma Cell Proliferation *In Vitro*

To understand the role of SAMMSON in melanoma, A375 and A875 were transfected with ASO to knock down SAMMSON expression. Knockdown efficiency was confirmed in A375 cells transfected with GapmeR3, GapmeR11, and NC. GapmeR3 had a higher knockdown efficiency (approximately 87%) at 48 h posttransfection than the control group (Figure 2(a)) and was chosen for subsequent experiments. The proliferation and clonogenicity of A375 and A875 cells were reduced after transfection with GapmeR3 (Figures 2(b)–2(e)).

Compared with the control group, SAMMSON knockdown decreased the relative mRNA expression of Bcl-2, CDK2, and CDK4 in A375 and A875 cells (Figures 2(g)–2(i)) and increased the mRNA expression of caspase 3 and P27 (Figures 2(f) and 2(j)). In addition, SAMMSON silencing decreased the protein levels of CDK4 and cyclin D1 in A375 cells (Figures 2(k) and 2(l)). These results confirm that SAMMSON promotes melanoma cell proliferation by regulating the expression of proliferation-associated genes.

### 3.3. SAMMSON Knockdown Inhibits Melanoma Cell Migration and Invasion *In Vitro*

The impact of SAMMSON expression on the migration and invasion of melanoma cells was evaluated using Transwell assays. Compared with the control groups, SAMMSON silencing significantly decreased the migration and invasion of A375 and A875 cells (Figures 3(a) and 3(b)). Moreover, SAMMSON knockdown reduced the mRNA expression of EMT-related genes, including vimentin (Figure 3(d)), N-cadherin (Figure 3(e)), MMP9 (Figure 3(f)), and MMP2 (Figure 3(g)). In contrast, SAMMSON silencing increased E-cadherin mRNA expression (Figure 3(c)). Western blots showed that knockdown decreased the protein expression of MMP9 and MMP2 (Figures 3(h) and 3(i)). These results reveal that SAMMSON promotes melanoma cell migration and invasion by regulating the expression of factors involved in EMT and MMPs.

### 3.4. SAMMSON Reduces FOXA2 Protein Expression

To further investigate the genes regulated by SAMMSON, a total of 613 differentially expressed genes (DEGs) between patients with high (*n* = 150) and low (*n* = 155) expressions of SAMMSON were identified, which are shown with volcano plots (Figure 4(a)). Patient characteristics are shown in Table 4. Of these DEGs, 34 DEGs encoded TFs and were downregulated in patients with high SAMMSON expression (Figure 4(b)). Top eight downregulated TFs are listed in Table 5. The relative mRNA levels of FOXA2 were obviously downregulated in different melanoma cell lines compared with ELF and TCF21 (Figures 4(c)–4(e)). Western blots showed that SAMMSON knockdown increased FOXA2 protein levels in melanoma cells (Figure 4(f)), indicating that FOXA2 expression was regulated by SAMMSON. In addition, SAMMSON silencing decreased the expression levels of enhancer of zeste homolog 2 (EZH2) and methylated histone H3 in melanoma cells (Figures 4(g) and 4(h)).

### 3.5. FOXA2 Is Downregulated in Melanoma Tissues

The expression of FOXA2 in nevi and melanoma tissues was evaluated by immunohistochemistry (IHC) and calculation of IRSs. The results showed that FOXA2 protein was predominantly located in the nucleus of nevi cells and the cytoplasm of melanoma cells (Figure 5(a)). We found that 100% (11/11) of nevi samples had higher expression of FOXA2 in the nucleus, but only 8.9% (6/67) of melanoma samples had higher expression of FOXA2 in the cytoplasm (Figures 5(b) and 5(c)). Furthermore, IRS was significantly higher in the nucleus of nevi cells but similar across the cytoplasm of nevi and melanoma cells (Figures 5(d) and 5(e)). These results suggest that FOXA2 protein expression was markedly lower in melanoma than in nevi tissues.

### 3.6. FOXA2 Overexpression Inhibits Melanoma Cell Proliferation *In Vitro* and *In Vivo*

To determine the functions of FOXA2 in melanoma, we successfully established stable FOXA2-overexpressing A375 and A875 cells, which were verified by RT-qPCR and western blotting (Figures 6(a) and 6(b)). Confocal microscopy showed that FOXA2 immunostaining intensity was markedly enhanced in the nucleus of FOXA2-OE melanoma cells (Figures 6(c) and 6(d)). In addition, FOXA2-OE melanoma cells were more cohesive and spatially organized than control cells (Figures 6(e) and 6(f)).

Ectopic FOXA2 expression reduced cell proliferation and clonogenicity (Figures 7(a) and 7(b)). These results agree with the cell cycle analysis data demonstrating that the progression from G_0_/G_1_ to G_2_/M and S was inhibited in FOXA2-OE melanoma cells (Figure 7(c)). FOXA2 decreased the mRNA expression of genes involved in melanoma cell proliferation, including CDK2, CDK4, and cyclin D1 (Figures 7(d)–7(f)). Moreover, FOXA2 overexpression decreased the protein levels of CDK4 (Figure 7(g)) and increased the levels of P27 and P53 (Figures 7(h) and 7(i)), suggesting that FOXA2 suppresses melanoma cell proliferation by regulating the expression of cell cycle-related genes *in vitro*.

The effect of FOXA2 on tumor growth was assessed using a mouse xenograft model. Tumors derived from A375 FOXA2-OE cells developed more slowly than those from control cells (Figure 8(a)). Furthermore, tumor volume and mass were remarkably lower in the A375 FOXA2-OE group than in the control group (Figures 8(b) and 8(c)). These results suggest that FOXA2 inhibits melanoma cell proliferation *in vivo*.

### 3.7. FOXA2 Overexpression Inhibits Melanoma Cell Migration and Invasion *In Vitro*

Transwell assays were performed to evaluate the effect of FOXA2 expression on melanoma cell migration and invasion. The results showed that FOXA2 reduced the migration and invasion of A375 and A875 cells (Figures 9(a) and 9(b)). RT-qPCR and western blotting analyses indicated that FOXA2 overexpression increased E-cadherin expression levels and decreased the expression levels of vimentin, N-cadherin, and MMP2 in these cells (Figures 9(c)–9(j)). In addition, FOXA2 overexpression decreased the mRNA and protein levels of MMP9 (Figures 10(a) and 10(b)), whereas FOXA2 knockdown had the opposite effect (Figures 10(c) and 10(d)). These results suggest that FOXA2 inhibited melanoma cell migration and invasion by manipulating the expression of EMT-related genes and MMPs.

## 4. Discussion

lncRNAs play crucial roles in melanoma pathogenesis [18]. The lncRNA SAMMSON is overexpressed in various cancers, including hepatocellular carcinoma [19], glioblastoma [20], and thyroid cancer [21]. We found that SAMMSON was highly expressed in skin melanoma cell lines but not in renal carcinoma cell lines and nontumorigenic cell lines, consistent with previous findings in uveal melanoma [22]. *BRAF* and *NRAS* are the common driver mutations in cutaneous melanoma [23], whereas *GNAQ* and *GNA11* are the frequently somatic mutations in uveal melanoma [24]. These findings indicate that SAMMSON is consistently expressed in most melanomas independent of the mutational status of tumors. Moreover, higher SAMMSON expression was associated with poor 10-year OS in patients with melanoma, in line with observations in gastric cancer [25]. The present study is the first to assess the correlation between SAMMSON expression and melanoma prognosis. However, larger studies are necessary to determine the prognostic value of SAMMSON in melanoma.

SAMMSON promotes cell viability by regulating mitochondrial function in both cutaneous melanoma [10] and uveal melanoma [22]. It was found that SAMMSON knockdown induced significant apoptosis in conjunctival melanoma cells [22], whereas the specific underlying mechanism is still unknown. Given that conjunctival melanoma has a higher genetic similarity with cutaneous melanoma [26], it is speculated that SAMMSON may increase conjunctival melanoma survival by maintaining mitochondrial homeostasis under the same mechanism, though further studies are still needed for confirmation. In contrast, we showed that SAMMSON expression was positively correlated with the expression of CDK2, CDK4, and cyclin D1. In line with our observations, Han et al. revealed that the P53 expression was significantly elevated in SAMMSON-silenced melanoma cells [27]. These findings indicated that SAMMSON has influence on melanoma cell proliferation by regulating the expression of cell cycle proteins. Nonetheless, the molecular mechanisms through which SAMMSON regulates cell cycle molecules need to be further investigated.

SAMMSON is highly expressed in lymph node metastases from patients with oral mucosal melanoma [28], suggesting that SAMMSON overexpression contributes to melanoma metastasis. In line with this observation, we found that SAMMSON expression was higher in metastatic skin melanoma tissues than in primary tumors. Furthermore, SAMMSON knockdown reduced the migration and invasion of melanoma cells, in agreement with previous findings in liver cancer cells [29].

EMT is implicated in carcinogenesis and confers metastatic properties to cancer cells by enhancing cell mobility and invasion [30, 31]. A study suggested that MMPs were involved in EMT [32]. lncRNAs promoted EMT by regulating the expression of EMT-related genes, such as Snail, Slug, and Twist in colorectal cancer [33] and prostate cancer [34]. SAMMSON silencing reduced the invasive ability of glioblastoma cells by upregulating E-cadherin and downregulating N-cadherin [20]. Nonetheless, little is known about the effect of SAMMSON on MMP expression. We found that SAMMSON knockdown downregulated MMP2 and MMP9 expressions in melanoma cells, implying that SAMMSON promotes melanoma cell migration and invasion by regulating EMT and MMPs. However, the effect of SAMMSON on MMP expression in melanoma and the mechanisms by which SAMMSON regulates EMT are incompletely understood.

FOXA2 expression was decreased in melanoma cell lines and tissues, consistent with the findings in gastric cancer [35] and liver cancer [36]. Previous research demonstrated that FOXA2 suppressed the survival of melanoma by inhibiting melanoma tumor stem cells [37]. However, we found that FOXA2 overexpression inhibited G_1_/S phase transition by regulating the expression of cell cycle-related proteins. Jang et al. showed that FOXA2 activated Bax and P21 gene transcription by binding to the promoter region of genes in non-small-cell lung cancer cells [13]. In line with our observations, FOXA2 was reported to inhibit melanoma cell migration and invasion [14], while the exact molecular mechanism was not fully elucidated. In this study, we found that FOXA2 regulates the expression of EMT molecules, which have been well studied in other tumors [38, 39], but rarely reported in melanoma. Surprisingly, we demonstrated for the first time in melanoma cells that FOXA2 represses the gene transcription of MMP9 and MMP2.

FOXA2 is involved in cancer pathogenesis and is targeted by noncoding RNAs. For instance, miR-942 inhibits breast cancer cell proliferation, migration, and invasion by downregulating FOXA2 expression [40], and FTX suppresses lung cancer proliferation and metastasis by upregulating FOXA2 [41]. Consistent with these observations, we found that SAMMSON silencing induced FOXA2 expression in different melanoma cell lines. Hence, we explore the possible relationship between SAMMSON and FOXA2.

The trimethylation of lysine 27 in histone H3 (H3K27me3) leads to gene silencing in prostate cancer [42]. Lu et al. found that EZH2 inhibited FOXA2 transcription in mouse bone marrow mesenchymal stem cells by increasing the H3K27me3 level of the FOXA2 promoter [43]. EZH2 is the catalytically active subunit of polycomb repressive complex 2, which decreases gene expression by regulating the expression level of H3K27me3 and plays an important role in tumorigenesis [44, 45]. These findings suggest that FOXA2 gene expression is regulated by H3K27me3 modification mediated by EZH2. lncRNAs regulate tumorigenesis and tumor progression by interacting with EZH2. For instance, LINC-PINT inhibited melanoma proliferation and migration by binding to EZH2 [46], and lncRNA-BLACAT1 promoted pancreatic cancer cell proliferation and migration by suppressing CDKN1C expression via EZH2-induced H3K27me3 [47].

In our study, SAMMSON knockdown decreased the expression level of EZH2 and H3K27me3 in melanoma cells, suggesting that SAMMSON modulates FOXA2 expression by regulating the EZH2/H3K27me3 axis. Nevertheless, further studies are warranted to elucidate the mechanism governing the interaction between these factors. Furthermore, another study is being underway to assess the regulation of FOXA2 by SAMMSON and the modulation of MMP9 expression by FOXA2.

## 5. Conclusion

SAMMSON was significantly upregulated in melanoma and promoted cancer progression by inhibiting FOXA2 expression. To the best of our knowledge, this study is the first to assess the association between SAMMSON and FOXA2 expression in melanoma. Given that mortality rates tend to be higher in the late stage of melanoma, SAMMSON-targeted therapies are promising for melanoma.

## Figures and Tables

**Figure 1:** lncRNA SAMMSON is upregulated in human melanoma tissues and cell lines, and lower SAMMSON expression is associated with increased 10-year OS. (a) Analysis of the GEPIA database on the relative SAMMSON expression in melanoma tissue and normal tissue (^∗^*p* < 0.05, Mann–Whitney *U* test). (b) Analysis of the GEO database on SAMMSON expression in normal skin tissues, primary tumors, and metastatic melanoma tissues (^∗∗^*p* < 0.01, ^∗∗∗^*p* < 0.001, Mann–Whitney *U* test). (c) Analysis of the TCGA database on SAMMSON expression in primary tumors and metastatic tissues (^∗^*p* < 0.05, Mann–Whitney *U* test). (d) RT-qPCR analysis of SAMMSON expression in melanoma tissues and normal adjacent tissues (^∗^*p* < 0.05, ^∗∗^*p* < 0.01, and ^∗∗∗^*p* < 0.001, paired *t*-test). (e) RT-qPCR analysis of SAMMSON expression in human melanoma cell lines (SK-MEL-110, A375, A875, SK-MEL-28, and M21) and human renal carcinoma cell lines (ACHN, CaKi-1, and 786-O). The immortalized human keratinocyte cell line HaCaT and proximal tubule epithelial cell line HK-2 were used as controls. (f) Kaplan-Meier OS curves for patients with MM from the GSE19234 dataset (*p* = 0.0073, log-rank test).

**Figure 2:** SAMMSON silencing inhibits melanoma cell proliferation *in vitro*. (a) The knockdown efficiency of the ASO-mediated suppression of SAMMSON in A375 cells was detected by RT-qPCR. (b, c) Cell growth curves of SAMMSON knockdown and control melanoma cells were plotted using MTT assays. The horizontal coordinate represents the time of cell culture, and the ordinate represents the absorbance value of the cell at the wavelength of 490 nm. (d, e) Evaluation of the proliferative capacity of SAMMSON-silenced and control melanoma cells using the colony formation assay. (f–j) RT-qPCR analysis of the relative mRNA expression of caspase 3, Bcl-2, CDK2, CDK4, and P27 in SAMMSON-silenced and control melanoma cells. (k, l) Western blotting analysis of the protein expression of CDK4 and cyclin D1 in SAMMSON-silenced and control melanoma cells. ^∗^*p* < 0.05, ^∗∗^*p* < 0.01, ^∗∗∗^*p* < 0.001, and ^∗∗∗∗^*p* < 0.0001 vs. control cells.

**Figure 3:** SAMMSON silencing inhibits melanoma cell migration and invasion *in vitro*. (a, b) Analysis of the effect of SAMMSON knockdown on melanoma cell migration and invasion using Transwell assays. Representative images of migrated and invaded cells are shown in the top panel; quantitative results are shown below the images. (c–g) RT-qPCR analysis of the relative mRNA expression of E-cadherin, vimentin, N-cadherin, MMP9, and MMP2 in SAMMSON-silenced and control melanoma cells. (h, i) Western blotting analysis of the protein expression of MMP9 and MMP2 in SAMMSON-silenced and control melanoma cells. Scale bars = 100 *μ*m. ^∗^*p* < 0.05, ^∗∗^*p* < 0.01, ^∗∗∗^*p* < 0.001, and ^∗∗∗∗^*p* < 0.0001 vs. control cells.

**Figure 4:** SAMMSON inhibits FOXA2 protein expression in melanoma cells. (a) Volcano plot of differentially expressed genes in patients with high and low SAMMSON expression. Red, green, and black indicate upregulated, downregulated, and unaffected genes, respectively. (b) Venn diagram for the TFs in DEGs. (c–e) RT-qPCR analysis of the relative mRNA expression of TCF21, FOXA2, and ELF5 in HaCaT and melanoma cell lines. (f) Western blotting analysis of the protein expression of FOXA2 in SAMMSON-silenced and control melanoma cells. (g) RT-qPCR analysis of the relative mRNA expression of EZH2 in SAMMSON-silenced and control melanoma cells. (h) Western blotting analysis of the protein expression of EZH2 and H3K27me3 in SAMMSON-silenced and control melanoma cells. ^∗∗^*p* < 0.01 vs. control cells.

**Figure 5:** Immunohistochemical staining of FOXA2 in nevi and melanoma tissues. (a) Representative images of IHC staining for FOXA2 in nevi (*n* = 11) and melanoma (*n* = 67). FOXA2 staining was stronger in nevi cells and was located mainly in the nucleus. Staining was weaker in melanoma tissues and was located primarily in the cytoplasm. (b, c) Percentage of nevi and melanoma tissues with high or low FOXA2 expression in the cytoplasm and nucleus. (d, e) IRSs of FOXA2 staining in nevi and melanoma tissues. Scale bars = 20 *μ*m. ^∗^*p* < 0.05, ^∗∗∗∗^*p* < 0.0001.

**Figure 6:** Establishment and identification of FOXA2 overexpression in melanoma cell lines. (a) RT-qPCR analysis of the relative mRNA expression of FOXA2 in NC-OE and FOXA2-OE melanoma cells. (b) Western blotting analysis of the protein expression of FOXA2 in NC-OE and FOXA2-OE melanoma cells. (c, d) Representative images of immunofluorescence staining for FOXA2 in NC-OE and FOXA2-OE melanoma cells. (e, f) Representative figures show that FOXA2-OE melanoma cells were more cohesive and spatially organized than NC-OE cells. Scale bars = 50 *μ*m. ^∗∗∗^*p* < 0.001, ^∗∗∗∗^*p* < 0.0001 vs. control cells.

**Figure 7:** FOXA2 inhibits melanoma cell proliferation *in vitro*. (a) Cell growth curves of NC-OE and FOXA2-OE melanoma cells were plotted using MTT assays. (b) The proliferative capacity of NC-OE and FOXA2-OE melanoma cells was determined by plate clone formation assays. (c) Flow cytometry analysis of the cell cycle of NC-OE and FOXA2-OE melanoma cells. (d–f) RT-qPCR analysis of the relative mRNA expression of CDK2, CDK4, and cyclin D1 in NC-OE and FOXA2-OE melanoma cells. (g–i) Western blotting analysis of the protein expression of CDK4, P27, and P53 in NC-OE and FOXA2-OE melanoma cells. ^∗^*p* < 0.05, ^∗∗^*p* < 0.01, ^∗∗∗^*p* < 0.001, and ^∗∗∗∗^*p* < 0.0001 vs. control cells.

**Figure 8:** FOXA2 inhibits subcutaneous melanoma xenograft growth in mice. (a) Nude mice (*n* = 5) were injected subcutaneously with A375 NC-OE and A375 FOXA2-OE melanoma cells. After 21 days, mice were sacrificed, and tumors were collected. (b) Tumor size was measured on different days postinjection and expressed as volume (mm^3^) (^∗∗^*p* < 0.01, ^∗∗∗^*p* < 0.001 vs. the control, two-way analysis of variance). (c) Tumor weights in the A375 NC-OE and A375 FOXA2-OE groups were measured after tumor samples were harvested. ^∗∗∗^*p* < 0.001 vs. the control group.

**Figure 9:** FOXA2 inhibits melanoma cell migration and invasion *in vitro*. (a, b) Analysis of the effect of FOXA2 on melanoma cell migration and invasion using Transwell assays. Quantitative results are shown below the images. (c–f) RT-qPCR analysis of the relative mRNA expression of E-cadherin, vimentin, N-cadherin, and MMP2 in NC-OE and FOXA2-OE melanoma cells. (g–j) Western blotting analysis of the protein expression of E-cadherin, vimentin, N-cadherin, and MMP2 in NC-OE and FOXA2-OE melanoma cells. Scale bars = 100 *μ*m. ^∗^*p* < 0.05, ^∗∗^*p* < 0.01, ^∗∗∗^*p* < 0.001, and ^∗∗∗∗^*p* < 0.0001 vs. control cells.

**Figure 10:** FOXA2 inhibits MMP9 transcription. (a, b) RT-qPCR and western blotting analyses of the mRNA and protein expression of MMP9 in NC-OE and FOXA2-OE melanoma cells. (c, d) RT-qPCR and western blotting analyses of the mRNA and protein expression of MMP9 in control and FOXA2-silenced melanoma cells. ^∗∗^*p* < 0.01, ^∗∗∗^*p* < 0.001, and ^∗∗∗∗^*p* < 0.0001 vs. control cells.

**Table 1:** Clinicopathologic characteristics of patients with malignant melanoma from the MME1004i tissue microarray database.

Characteristics	*n* (%)
*Gender*	
Male	39 (58.2%)
Female	28 (41.8%)
Age (years)	
<60	39 (58.2%)
≥60	28 (41.8%)
*Lymph node metastasis*	
N0	51 (76.2%)
N1-4	8 (11.9%)
Not available	8 (11.9%)
*Distant metastasis*	
M0	58 (86.6%)
M1	1 (1.5%)
Not available	8 (11.9%)
*Maximum tumor diameter (cm)*	
<4	11 (36.5%)
≥4	48 (63.5%)
Not available	8 (11.9%)
*TNM stage*	
I/II	38 (56.7%)
III/IV	5 (7.5%)
Not available	24 (35.8%)

**Table 2:** Clinicopathologic parameters of patients with malignant melanoma from the datasets GSE15605 and GSE19234.

Characteristics	GSE15605			GSE19234
	Normal	Primary	Metastatic	
Gender				
Male	13 (81.2%)	32 (69.6%)	6 (50%)	28 (63.6%)
Female	3 (18.8%)	14 (30.4%)	6 (50%)	16 (36.4%)
Age (years)				
≥60	5 (31.2%)	23 (50%)	6 (50%)	19 (43.2%)
<60	11 (68.8%)	23 (50%)	6 (50%)	25 (56.8%)
Diagnosis				
Superficial spreading melanoma		28 (60.9%)	8 (66.7%)	
Desmoplastic melanoma		1 (2.2%)	2 (16.7%)	
Acral lentiginous melanoma		3 (6.5%)	2 (16.7%)	
Mucosal melanoma		0	0	
Lentigo maligna melanoma		1 (2.2%)	0	
Nodular melanoma		8 (17.4%)	0	
Other types		5 (10.9%)	0	
Mutation				
WT				
BRAF		20 (43.5%)	8 (66.7%)	
NRAS		6 (13.0%)	2 (16.7%)	
Stage				
IIIA				4 (9.0%)
IIIB				23 (52.3%)
IIIC				12 (27.3%)
IV				5 (11.4%)

BRAF: V-RAF murine sarcoma viral oncogene homolog B1; NRAS: neuroblastoma-rat sarcoma viral oncogene homolog.

**Table 3:** The sequences of all primers.

Gene	Primer sequence	Product length (base pairs)
SAMMSON	F: 5′-CCTCTAGATGTGTAAGGGTAGT-3′	278
	R: 5′-TTGAGTTGCATAGTTGAGGAA-3′	

FOXA2	F: 5′-GGAACACCACTACGCCTTCAAC-3′	134
	R: 5′-AGTGCATCACCTGTTCGTAGGC-3′	

EZH2	F: 5′-GACCTCTGTCTTACTTGTGGAGC-3′	115
	R: 5′-CGTCAGATGGTGCCAGCAATAG-3′	

MMP9	F:5′-GCCACTACTGTGCCTTTGAGTC-3′	125
	R:5′-CCCTCAGAGAATCGCCAGTACT-3′	

MMP2	F: 5′-AGCGAGTGGATGCCGCCTTTAA-3′	138
	R: 5′-CATTCCAGGCATCTGCGATGAG-3′	

E-cadherin	F: 5′-GCCTCCTGAAAAGAGAGTGGAAG-3′	131
	R: 5′-TGGCAGTGTCTCTCCAAATCCG-3′	

N-cadherin	F: 5′-CCTCCAGAGTTTACTGCCATGAC-3′	149
	R: 5′-GTAGGATCTCCGCCACTGATTC-3′	

Vimentin	F: 5′-AGGCAAAGCAGGAGTCCACTGA-3′	100
	R: 5′-ATCTGGCGTTCCAGGGACTCAT-3′	

Caspase 3	F: 5′-GAAATTGTGGAATTGATGCGTGA-3′	164
	R: 5′-CTACAACGATCCCCTCTGAAAAA-3′	

Cyclin D1	F: 5′-GCTGCGAAGTGGAAACCATC-3′	135
	R: 5′-CCTCCTTCTGCACACATTTGAA-3′	

CDK2	F: 5′-CCAGGAGTTACTTCTATGCCTGA-3′	90
	R: 5′-TTCATCCAGGGGAGGTACAAC-3′	

CDK4	F: 5′-TCAGCCAGCTTGACTGTTCCA-3′	94
	R: 5′-GCCTAGATTTCCTTCATGCCA-3′	

P27	F: 5′-ATAAGGAAGCGACCTGCAACCG-3′	119
	R: 5′-TTCTTGGGCGTCTGCTCCACAG-3′	

Bcl-2	F: 5′-GTGCCTGCTTTTAGGAGACCGA-3′	128
	R: 5′-GAGACCACACTGCCCTGTTGATC-3′	

Bax	F: 5′-AGACACTCGCTCAGCTTCTTG-3′	116
	R: 5′-CTTTTGCTTCAGGGTTTCATC-3′	

*β*-Actin	F:5′-GGATTACCCTGAAATGGGCTTGT-3′	102
	R:5′-CTCTGAGGTTAGCTGCATCGACAT-3′	

GAPDH	F: 5′-GTCTCCTCTGACTTCAACAGCG-3′	131
	R: 5′-ACCACCCTGTTGCTGTAGCCAA-3′	

**Table 4:** Clinicopathologic parameters in skin cutaneous melanoma patients from the TCGA database.

Characteristics	*n* (%)
*Gender*	
Male	180 (59%)
Female	125 (41%)
*Age*	
<60	159 (52.1%)
≥60	146 (47.9%)
*T stage*	
T1-T2	77 (25.2%)
T3-T4	160 (52.5%)
Not available	68 (22.35)
*N-stage*	
N0	151 (49.5%)
N1, N2, and N3	140 (45.9%)
Not available	14 (4.6%)
*M-stage*	
M0	274 (89.8%)
M1	12 (3.9%)
Not available	19 (6.3%)
*Clinical stage*	
I/II	145 (47.5%)
III/IV	122 (40%)
Not available	38 (12.5%)

**Table 5:** Top eight downregulated transcription factors in skin cutaneous melanoma patients with high SAMMSON expression.

Gene	Protein name	Fold-change	*p* value
PRB4	Proline-rich protein BstNI subfamily 4	-8.57039978	0
PRH1	Proline-rich protein HaeIII subfamily 1	-6.001785093	5.52*E* − 165
KRT17	Keratin 17	-3.368087123	1.13*E* − 117
PRB1	Proline-rich protein BstNI subfamily 4	-5.642715435	2.12*E* − 104
TCF21	Transcription factor 21	-4.451119203	2.51*E* − 71
MKX	Mohawk homeobox	-3.332287746	1.15*E* − 43
FOXA2	Forkhead box A2	-3.927396483	6.98*E* − 38
ELF5	E74-like ETS transcription factor 5	-3.054746206	2.56*E* − 30

## Data Availability

The datasets analyzed in this study can be found in the GEO database (GSE15605 and GSE19234) and TCGA database. All data supporting this study are available from the corresponding author upon reasonable request.

## Abbreviations

lncRNA: Long noncoding RNA
SAMMSON: Survival-associated mitochondrial melanoma-specific oncogenic noncoding RNA
EMT: Epithelial-to-mesenchymal transition
MMPs: Matrix metalloproteinases
FOXA2: Forkhead box A2
MM: Malignant melanoma
TF: Transcription factor
IRS: Immunoreactive score
TCGA: The Cancer Genome Atlas
GEO: Gene Expression Omnibus
DMEM: Dulbecco's modified Eagle's medium
PBS: Phosphate-buffered saline
ASO: Antisense oligonucleotide
OE: Overexpression
NC: Negative control
BSA: Bovine serum albumin
cDNA: Complementary DNA
OS: Overall survival
DEGs: Differentially expressed genes
EZH2: Enhancer of zeste homolog 2
IHC: Immunohistochemistry
H3K27me3: Trimethylation of lysine 27 in histone H3.
